The article "Molecular diagnosis and characterization of Cryptosporidium spp. in turkeys and chickens in Germany reveals evidence for previously undetected parasite species" was published in 2017. Journal: PLoS One.

# Molecular diagnosis and characterization of *Cryptosporidium* spp. in turkeys and chickens in Germany reveals evidence for previously undetected parasite species

**DOI:** 10.1371/journal.pone.0177150

**Published:** 2017-06-02

**Authors:** Yosra A. Helmy, Jürgen Krücken, El-Sayed M. Abdelwhab, Georg von Samson-Himmelstjerna, Hafez M Hafez

**Affiliations:** 1 Food Animal Health Research Program, Department of Veterinary Preventive Medicine, Ohio Agricultural Research and Development Center, Ohio State University, Wooster, Ohio, United States of America; 2 Department of Animal Hygiene, Zoonoses and Animal Ethology, Faculty of Veterinary Medicine, Suez Canal University, Ismailia, Egypt; 3 Institute for Parasitology and Tropical Veterinary Medicine, Freie Universität Berlin, Berlin, Germany; 4 Institute of Molecular Biology, Friedrich-Loeffler-Institute, Federal Research Institute for Animal Health, Greifswald-Insel Riems, Germany; 5 Institute of Poultry Diseases, Freie Universität Berlin, Berlin, Germany; Utah State University, UNITED STATES

## Abstract

A total of 256 fecal specimens were randomly collected from farmed poultry in Germany and screened for the presence of *Cryptosporidium* spp. by PCR and further characterized by direct automated DNA sequencing. Using a nested PCR amplifying approximately 830 bp 18S rDNA fragment, 7.03% (n = 18) of the samples were *Cryptosporidium*-positive. In detail, *Cryptosporidium* was detected in 9.3% (8/86) of turkeys, 5.7% (9/158) of broilers and 8.3% (1/12) of layers. After DNA sequencing, *Cryptosporidium parvum* the most frequently observed species was identified in 5.1% (13/256) of all poultry species, including 8.1% (7/86) of turkeys, 3.2% (5/158) of broilers and 8.3% (1/12) of layers. *Cryptosporidium baileyi* was detected in 1.3% (2/256) of the broilers only. Three novel unclassified *Cryptosporidium* spp. were detected in 1.2% (1/86) of turkeys and 1.3% (2/158) of broilers. The infection rate was high in 13–20 week old turkeys, 1–6 weeks old broilers and >20 weeks old layers but differences between age groups were not significant. This is the first study in Germany uses molecular methods for the detection of *Cryptosporidium* in poultry. The results indicate that *Cryptosporidium* parasites are common among broilers and turkeys in Germany. Considering the large size of the poultry industry, the large amount of poultry meat that is consumed and the fact that *C*. *parvum* is also the most common *Cryptosporidium* parasite in humans, poultry might also be a source of human infections.

## Introduction

*Cryptosporidium* are among the most prevalent enteric protozoan parasites that infect a wide range of host species, including mammals, birds, reptiles and fish [1,2]. In birds, cryptosporidiosis was first described in the caeca of chicken by Tyzzer [3]. Birds are considered a reservoir for human infections due to the possible transmission of *Cryptosporidium parvum* [4] and frequent human infections with *Cryptosporidium meleagridis* [5,6]. *Cryptosporidium* has been reported in more than 30 avian species worldwide, including chickens, turkeys, ducks, geese, quails, pheasants and peacocks [2,7]. However, there were only a few studies that have examined the genetic diversity of *Cryptosporidium* spp. among avian hosts. *Cryptosporidium* are transmitted through ingestion or inhalation of sporulated oocysts in contaminated materials, contaminated litter, feces, water and dust. Poor hygienic conditions have been associated with increased prevalence of the disease in poultry flocks [4].

Cryptosporidiosis in chickens and/or turkeys is usually caused by *C*. *baileyi* and *C*. *meleagridis*, [8] and rarely *C*. *parvum* [9] and *Cryptosporidium galli* [10]. *C*. *baileyi*, which is generally the most prevalent species in domestic poultry, causes respiratory and intestinal infections (including histopathological changes in the bursa of Fabricius) [11,12], whereas *C*. *meleagridis* infects the intestines causing mild to severe diarrhea [13]. *C*. *parvum* and *C*. *galli* infect chickens or turkeys without showing clinical signs [10,14]. Birds-to-human transmission of *C*. *meleagridis* has been frequently reported in humans, particularly involving immune-compromised patients and children [15]. Moreover, the reverse zoonotic transmission (from human-to-animals) of *C*. *parvum*, the most prevalent cryptosporidium in humans and farm animals, has been also reported [16].

In the present study, fecal samples obtained from 256 commercial chicken and turkey flocks in 2013/2014 in Germany were examined for *Cryptosporidium* using PCR. *Cryptosporidium* strains detected in this study were genetically characterized to gain a better understanding of the distribution of *Cryptosporidium* spp. in chickens and turkeys and the genetic relationship to other *Cryptosporidium* spp. in animals and humans.

## Materials and methods

### Ethics statement

All samples were collected from poultry farms. Therefore, no ‎endangered species were involved. Since faecal samples were collected after ‎natural defecation of the animals from the floor, no permission regarding laws ‎on animal protection was required. We have received permission from the farm owners to collect the samples. Samples were taken by the animal owners ‎and sent to the Institute of Poultry Diseases, Freie Universität Berlin.

### Sample collection

Fresh pool faecal samples were collected from 256 poultry flocks kept on the floor in Germany at different ages between February 2013 and August 2014 (S1 Table). Each sample contained 20–30 single faecal droppings from different areas inside the poultry house that were pooled into a single sample. In total 86 samples from fattening turkey flocks, 158 pool samples from broiler flocks, and 12 pool samples from layer flocks were collected. All samples were collected from apparently healthy flocks in the frame of the *Salmonella* surveillance program and proved to be free of *Salmonella*. Samples were transferred to the Institute of Parasitology and Tropical Veterinary Medicine, Berlin, Germany and stored at -20°C until examination. All samples were examined by nested PCR targeting the 18S rDNA and gp60 genes as described below.

### DNA extraction

DNA was extracted using the NucleoSpin Soil kit (Macherey-Nagel, Germany) and the extracted DNA was quantified on a Take3 plate (Biotek, Germany). DNA was stored at -20°C until use.

### Species identification by PCR

Identification of Cryptosporidium species was performed essentially as described previously (Ref Helmy et al Vet Parasitol) with minor modifications. Initially, a 1325 bp fragment of the 18S small subunit ribosomal DNA (18S rDNA) gene was amplified out using the primers 5′-TTCTAGAGCTAATACATGCG-3′ and 5′-CCCTAATCCTTCGAAACAGGA-3′. Then, a nested PCR using the primers 5′-GGAAGGGTTGTATTTATTAGATAAAG-3′ and 5′-AAGGAGTAAGGAACAACCTCCA-3′ aimed to obtain a 830 bp amplicon [17,18]. Both PCRs used 20 μl 1×HF buffer containing 0.02 U/μl Phusion Hot Start II DNA polymerase (Finnzymes), 0.25 μM of each primer and 0.2 mM of each dNTP. PCRs were performed on C1000 or S1000 PCR cyclers (Bio-Rad) using a temperature profile with an initial denaturation at 98°C for 30 s, followed by 40 cycles denaturation at 98°C for 10 s, annealing at 55°C for 30 s and elongation at 72°C for 30 s and a final extension at 72°C for 10 min. In the nested PCR 45 cycles were performed and the annealing temperature was set to 61.4°C [19].

### Sequence and phylogenetic analyses

PCR products were purified from 1.5% (wt/vol) agarose gels using Qiaquick PCR purification kit (Qiagen, Hilden, Germany) and sequenced by GATC Biotech (Germany). The obtained sequences were submitted to a BLAST search [20] to initially define the species and to further confirm the high similarity with other known sequences of *Cryptosporidium* spp. in GenBank. Phylogenetic relatedness of *Cryptosporidium* spp. detected in this study to other *Cryptosporidium* from animals and humans was analyzed by retrieving relevant gene sequences from GenBank database. Multiple sequence alignment was performed with MAFFT using the auto strategy selection [21] and edited by BioEdit version 7.1.7 [22]. Phylogenetic trees were generated using two sets of 18S rDNA gene sequences of Cryptosporidia. A tree was firstly constructed using 1232 out of 1391 gene sequences after removal of duplicates. Then, 70 gene sequences were selected including sequences generated in this study. A mid-point rooted tree was generated based on the best fit substitution model (GTR+ G) predicted by jModelTest 2.1.10 [23] using MrBayes as implemented in Topali v.2 [24]. A Bayesian tree was constructed with two independent runs each with 1,000,000 generations of MCMC simulations and a burn-in of 100,000. The phylogenetic tree was further edited by FigTree 1.4.2 (http://tree.bio.ed.ac.uk/) and Inkscape 2.0 (Free Software Foundation, Inc., Boston, USA).

### Statistical analysis

Statistical analysis was performed using mid-P exact probability tests and differences were considered significant when *p*-values ≤ 0.05 were obtained in OpenEpi software (http://www.openepi.com/Menu/OE_Menu.htm). Prevalence rates with 95% confidence intervals (CI) in poultry samples as identified by PCR were calculated as Wilson (score) intervals in OpenEpi Logistic regression analyses were performed using the glm command in R 3.3.1 software and considered the variables type of poultry (broiler, layer, turkey), the age group and the sex (male, female, mixed) as well as the geographical origin in terms of the German federal state in which the flock was located. The drop1 function was used to identify variables that could be eliminated from the model to improve (lower) the Akaike information criterion (AIC).

## Results

### Prevalence of *Cryptosporidium* spp.

The overall prevalence of *Cryptosporidium* spp. on the flock level was 7.0% (18/256) as estimated using the 18S rDNA PCR. The prevalence was 9.3% (8/86) in turkeys, 5.7% (9/158) in broilers and 8.3% (1/12) in layers (Table 1). However, the number in layers should be carefully considered due to the low number of tested flocks and the very wide 95% CI (1.5%–35.4%).

**Table 1:** Prevalence of *Cryptosporidium* spp. in different poultry species.

	Total number of flocks	*C*. *baileyi*	*C*. *parvum*	New *Cryptosporidium* genotypes	Total
		No. positive	No. positive	No. positive	No. positive
		(%)	(%)	(%)	(%)
		(95% CI^a^)	(95% CI)	(95% CI)	(95% CI)
Turkeys	86	0	7	1	8
		(0%)	(8.1%)	(1.2%)	(9.3%)
		(0–4.3%)	(4.0–15.9%)	(0.2–6.3%)	(4.8–17.3%)
Broilers	158	2	5	2	9
		(1.3%)	(3.2%)	(1.3%)	(5.7%)
		(0.3–4.5%)	(1.2–6.9%)	(0.3–4.5%)	(3.0–10.5%)
Layers	12	0	1	0	1
		(0%)	(8.3%)	(0%)	(8.3%)
		(0–22.1%)	(1.5–35.4%)	(0–22.1%)	(1.5–35.4%)
Total	256	2	13	3	18
		(0.8%)	(5.1%)	(1.2%)	(7.0%)
		(0.2–2.8%)	(3.0–8.1%)	(0.4–3.4%)	(4.5–10.8%)

^a^95% confidence interval.

### Age patterns of *Cryptosporidium* in fattening turkeys

The prevalence rates of *Cryptosporidium* infection in turkeys were 13.8% (4/29) between week 13 to 20 showing a prevalence of while the prevalence in broilers between weeks 1 to 6 was 5.7% (9/158) and 8.3% (1/12) in layers more than 20 weeks of age (Table 2).

**Table 2:** Age distribution in relation to detected *Cryptosporidium* spp. in different poultry species.

	Turkey	Broiler	Layers	Total
	No. positive	No. positive	No. positive	No. positive
	(%)	(%)	(%)	(%)
	(95% CI^a^)	(95% CI)	(95% CI)	(95% CI)
1–6 weeks	1/20	9/158	0.0	10/175
	(5%)	(5.7%)		(5.7%)
	(0.8–23.6)	(3.0–10.5)		(3.1–10.2)
7–12 weeks	0.0	0.0	0.0	0/17
				(0%)
				(0–18.4)
13–16 weeks	3/24	0.0	0.0	3/24
	(12.5%)			(12.5%)
	(4.3–31.0)			(4.3–31.0)
13–16 weeks	3/24	0.0	0.0	3/24
	(12.5%)			(12.5%)
	(4.3–31.0)			(4.3–31.0)
17–20 weeks	1/5	0.0	0.0	1/5
	(20%)			(20%)
	(3.6–62.4)			(3.6–62.4)
>20 weeks	0.0	0.0	1/12	1/12
			(8.3%)	(8.3%)
			(1.5–35.4)	(1.5–35.4)
Unknown	3/23	0.0	0.0	3/23
	(13%)			(13%)
	(4.5–32)			(4.5–32)
Total	8/86	9/158	1/12	18/256
	(9.3%)	(5.7%)	(8.3%)	(7.03%)
	(4.8–17.3)	(3.0–10.5)	(1.5–35.4)	(4.5–10.8)

### Potential effects of flock-associated variables on presence of *Cryptosporidium* sp.

Statistical analysis was hampered by the fact that sex and age were not useful variables for chicken flocks since variables were highly collinear. All broilers were male and 1–6 weeks old while all layers were female and older than 20 weeks. Pairwise mid-P exact tests revealed no significant differences (p>0.05) in the prevalence of *Cryptosporidium* spp. between broilers, layers and turkeys. For turkeys, exclusively male, exclusively female and mixed flocks were available. However, neither in pairwise mid-P exact tests nor in logistic regression analysis a significant effect of the sex could be identified. Turkey flocks belonged to all the age categories between 0 and 20 weeks (Table 2) but again no effect of the age on the probability of a flock to be positive for *Cryptosporidium* sp. was detected using mid-P exact tests or logistic regression analysis.

Logistic regression analysis with data for all types of poultry using the type of host (turkey, broilers and layers), the sex, the federal state as geographical variable and the age (in terms of weeks after hatching) did not reveal any significant effect of any of these variables on the chance to be positive for *Cryptosporidium* sp. Stepwise reduction of the model using the drop1 function in R to optimize the AIC also did not identify any variable with significant statistical effect. Comparable analyses were conducted separately for broilers and turkeys. Layers were excluded due to the small numbers of layer flocks. In the context of broilers and turkeys the breeding line was also included as additional variable. However, again no significant influence of any of the explanatory variables could be identified.

### Sequence and phylogenetic analysis of the 18S rDNA

Sequence analysis revealed the presence of *C*. *parvum*, *C*. *baileyi* and three genotypes that could not be allocated to any species. The overall prevalence of *C*. *parvum* was 5.1% (13/256). *C*. *parvum* was detected in 8.1% (7/86) of turkey and 3.2% (5/158) of broiler flocks and was the only species detected in layer flocks with 8.3% (1/12) (Table 1). *C*. *baileyi* was detected in 1.3% (2/158) of broilers. Three new unclassified *Cryptosporidium* genotypes (designated *C*. *avian* genotypes VII, VIII and IX) were detected in 1.2% (1/86) of turkeys and 1.3% (2/158) of broilers (Table 1). *C*. *parvum* was significantly more frequently found in all poultry flocks than *C*. *baileyi* (p = 0.004 in a mid-P exact test), any one of the three unclassified *Cryptosporidium* genotypes (p<0.001) or the three unclassified genotypes together (p = 0.011). However, it was not significantly more frequently observed than any of the other *Cryptosporidium* species/genotypes together (p = 0,059). For turkeys, *C*. *parvum* was more frequently found than *C*. *baileyi* (p = 0.007), any of the two unclassified genotypes (p = 0.035) but not for the two unclassified genotypes together (p = 0.101). Differences for broilers or layers alone were never significant.

A total of 786 nucleotides from 18S rDNA were successfully generated for each of 18 poultry flocks tested positive for *Cryptosporidium* sp. in this study. Sequences were submitted to the GenBank and assigned accession numbers (KX513529-KX513546). Phylogenetic relatedness of strains in this study is shown in Fig 1. All *C*. *parvum* strains in this study had 99.1% to 100% nucleotide identities with each other (Table 3). They clustered with human strains from patients in England, Slovenia, Spain, Czech, Japan, Egypt and Iran as well as animal strains from countries in all continents including *C*. *parvum* from a hedgehog in Germany (Fig 1). Two sequences (samples 99 and 224) clustered with *C*. *baileyi* isolated from birds and environmental water samples in Canada and China and they shared 99.6% nucleotide identity with each other. For the remaining three sequences, initially BLASTn searches using default parameters two had *C*. *baileyi* as best hits (samples 39 with 97.3%% identity and 165 with 97.7%% identity) while the remaining had *C*. *meleagridis* as best hit (sample 162 with 95.8% identity) but sequence identities were lower than in the intra-species clusters. Pairwise identities between these three sequences were 97.3–97.7% (Table 3). Phylogenetic analysis clustered all three sequences together although branch lengths were relatively long (Fig 1). Comparisons of branch lengths and pairwise sequence identities clearly show that these three sequences do not represent any of the *Cryptosporidium* sequences with 18S sequences deposited in GenBank. Therefore, these three new unclassified Cryptosporidium genotypes were designated as *Cryptosporidium* sp. broiler I and II (samples 162 and 165, respectively) and *Cryptosporidium* sp. turkey (sample 39) according to the host of origin as frequently done for unclassified *Cryptosporidium* genotypes.

**Fig 1:** Phylogenetic relationship of the 18S rDNA of *Cryptosporidium* strains detected in chickens and turkeys in Germany. A mid-point rooted tree was generated based on the best fit substitution model (GTR+G) predicted by jModelTest 2.1.10 [23] using MrBayes as implemented in Topali v.2 [24]. A Bayesian tree was constructed with two independent runs each with 1,000,000 generations of MCMC simulations and a 10% burn-in. The phylogenetic tree was further edited by FigTree 1.4.2 (http://tree.bio.ed.ac.uk/) and Inkscape 2.0 (Free Software Foundation, Inc., Boston, USA). Sequences generated in this study are written in blue.

**Table 3:** Nucleotide identity between 18S rDNA gene of *Cryptosporidium* genotypes detected from chickens and turkeys in Germany.

		*C*. *parvum*													*Cryptosporidium sp*.			*C*. *baileyi*	
															turkey	broiler 1	broiler 2		
Sample no.		7	3	42	61	87	13	86	24	116	118	205	20	135	39	162	165	99	224
***C*. *parvum***	**7**	ID	100	100	100	100	100	100	100	100	100	99.8	99.3	99.7	95.5	95.6	95.5	94.5	94.5
	**3**		ID	100	100	100	100	100	100	100	100	99.8	99.3	99.7	95.5	95.6	95.5	94.5	94.5
	**42**			ID	100	100	100	100	100	100	100	99.8	99.3	99.7	95.5	95.6	95.5	94.5	94.5
	**61**				ID	100	100	100	100	100	100	99.8	99.3	99.7	95.5	95.6	95.5	94.5	94.5
	**87**					ID	100	100	100	100	100	99.8	99.3	99.7	95.5	95.6	95.5	94.5	94.5
	**13**						ID	100	100	100	100	99.8	99.3	99.7	95.5	95.6	95.5	94.5	94.5
	**86**							ID	100	100	100	99.8	99.3	99.7	95.5	95.6	95.5	94.5	94.5
	**24**								ID	100	100	99.8	99.3	99.7	95.5	95.6	95.5	94.5	94.5
	**116**									ID	100	99.8	99.3	99.7	95.5	95.6	95.5	94.5	94.5
	**118**										ID	99.8	99.3	99.7	95.5	95.6	95.5	94.5	94.5
	**205**											ID	99.2	99.6	95.4	95.5	95.4	94.4	94.4
	**20**												ID	99.1	94.9	95.2	95	94	94
	**135**													ID	95.8	95.9	95.8	94.7	94.7
***C*. *turkey***	**39**														ID	97.3	97.3	95.6	95.4
***C*. *broiler***	**162**															ID	97.7	95.8	95.5
	**165**																ID	96.5	96.3
***C*.*baileyi***	**99**																	ID	99.6
	**224**																		ID

## Discussion

Birds are considered to be important disseminators of many pathogens worldwide. Due to their very wide host range, the protozoan parasites of the genus *Cryptosporidium* are of particular interest since some species can infect a wide variety of birds [2,4] and mammals including humans [25]. Despite of the importance of *Cryptosporidium* species identification for the understanding of the epidemiology of avian cryptosporidiosis, there are only a few studies that have tried molecular characterization of this protozoan in different poultry species. Currently, there are a only a few studies regarding chickens [4,26–28] and even less for turkeys [14,29].

In the present study, the overall prevalence of *Cryptosporidium* sp. was 7.0% and this result is not in agreement with a study that described a prevalence of *Cryptosporidium* in 5 fattening turkey flocks as well as one breeder flocks at several intervals in Germany [30]. In the latter, no *Cryptosporidium* infected flocks were identified using a traditional microscopical method which has a much lower sensitivity than nested PCR [31,32]. The new results from Germany are comparable with a recent report from China, where the prevalence detected by PCR was 10% in pooled samples collected between November 2010 and January 2012 from small groups of 5–7 around 90 days old broiler chickens [33].

In previous studies, the prevalence rates of *Cryptosporidium* sp. varied between different poultry species and different countries. In the present study, the prevalence was 9.3% in turkeys, 5.7% in broilers and 8.3% in layers. Using microscopical examination of the bursa and/or trachea, the infection rates in individual broilers in the European countries Scotland and Greece were 18.7% [34] and 24.3% [35], respectively. In Africa, using the same techniques, prevalence in broiler flocks was 37% in Morocco [36]. In Tunisia, 4.5% of individual broiler chickens were tested positive using the Ziehl Neelson staining of fecal smears [37]. Prevalences of 34% and 44% were observed in chickens and turkeys in Algeria using PCR analysis of samples taken from the Ileum [29]. In Asia, using histological examination, 36.8% of infection was observed in individual broilers and 33.3% in layers in Japan [38] while in Iran a rate of 23.8% was observed in broilers [39]. The overall infection rates with *Cryptosporidium* in China were reported to be 3.4% in broilers and 10.6% in layers chickens using bright-field microscopy of fecal samples after concentration of oocysts with the Sheather’s sugar flotation technique [27]. In Brazil, presence of *Cryptosporidium* DNA in feces was observed in 86% of the chickens using PCR [4]. The differences in prevalence rates observed might be attributed to the use of different detection methods (e.g. microscopic examination *vs*. PCR) and sample origin (tissue samples *vs*. feces). Moreover, differences in hygiene and management practices may also be responsible with low infection rates in birds related to efficient management and high infection rates related to poor hygiene, overpopulation and keeping different species of birds together [4,27,40].

The statistical analyses did not identify any factors that were associated with higher odds to be positive for *Cryptosporidium* spp. The main reason for this result is presumably the small number of positive flocks. The lack of an effect is particularly surprising regarding the age since *Cryptosporidium* infections in mammals are well not to particularly affect very young animals and decrease in prevalence and severity with increasing age [41]. Neither with the age as continuous variable in a logistic regression nor the use of age categories and comparison of prevalences between those categories with mid-p exact tests significant effects were identified. This might suggest that the effects of age on susceptibility to *Cryptosporidium* spp. differ between mammals and poultry.

In the present study, infection was detected in 13.8% of the turkey flocks in the age group of 13–20 weeks, in 5.7% of the 1–6 weeks old broiler flocks and in 8.3% of the >20 weeks old layer groups. These results were different from those obtained in China by Wang et al. [27] where in broiler chickens an individual infection rate of 4.9% was noted in birds aged from 1 to 20 days while in layer chickens an infection rate of 24.6% was observed in birds aged from 31 to 60 days. Also, infection was common in 4-9-week old turkeys in the USA [14]. The authors concluded that young birds were the most important risk group since their immune system is not yet fully developed. However, in the present study the infection of turkeys and layer chickens was in adult birds which may be due to stress factors, hence meat-turkeys are marketed around 20 weeks of age and egg production in layer chickens starts around 18 weeks of age.

In this study, *C*. *parvum* was the most prevalent species and was identified in broilers, layers and turkeys. *C*. *parvum* was also identified in chicks in Brazil [4] and turkeys in the USA [14]. The presence of DNA of *C*. *parvum* in the fecal samples of chickens and turkeys observed in the present study agrees with previous studies, where it was suggested that the birds would be acting as a source of infection and mechanical vectors, shedding oocysts in the environment, even if at a low rate [4,28,42,43].

*C*. *baileyi* is generally considered to be the most common species in domestic poultry with a widespread distribution in several hosts including chicken broilers and layers as well as turkeys causing worldwide considerable morbidity and mortality mainly due to respiratory disorders [8,33,44,45]. In contrast to the findings here where only two samples were positive for *C*. *baileyi*, *C*. *baileyi* was the predominant *Cryptosporidium* spp. in China in all age groups of chickens [27,33]. The detection rate of *C*. *parvum* in the present study is surprisingly significantly higher than the typical avian parasite *C*. *baileyi*. Sources for the infection of poultry with *C*. *parvum* in Germany remain to be elucidated. Contamination of water, feed and/or litter in poultry houses with oocysts from mammalian/human origin may be responsible.

Sequence and phylogenetic analyses indicated close relationship of the *C*. *parvum* strains in this study to isolates from human and animals, including the available *C*. *parvum* sequences from a hedgehog and a house mouse isolated from Germany. Whether chickens and turkeys screened in this study acquired the infection from humans and/or animals is unknown and further epidemiological investigations are required. Moreover, in the current study three new *Cryptosporidium* genotypes were identified with significant differences in their 18S rRNA sequences to all *Cryptosporidium* sequences deposited in the GenBank database. These three genotypes formed a separate, significant cluster in the phylogenetic tree. Sequences of other genes (e.g. *HSP70*, *gp60*, *COWP*) are required to properly position these genotypes in the *Cryptosporidium* phylogenetic tree using multi-locus phylogenetic analysis. Further morphological and host-specificity data would be required for a formal description of any new *Cryptosporidium* species represented by these genotypes.

## Conclusion

The present investigation revealed the presence of *C*. *parvum*, *C*. *baileyi* and three unclassified new *Cryptosporidium* genotypes in poultry in Germany. Further studies are required to understand the extent of zoonotic risks due to the frequent infection of poultry with *C*. *parvum* and the failure of gp60 PCRs to further genotype the parasites. In order to identify risk factors and sources of infection for the presence of cryptosporidiosis in poultry flocks a systematic comparison of prevalence rates between flocks under different management practices is needed. This should in particular include comparison of exclusively indoor- with free-range flocks.

## Supporting information

S1 Table Raw data for all poultry farms included in the study. (XLSX)
